# Early physical rehabilitation vs standard care for intracerebral hemorrhage stroke: A protocol for systematic review and meta-analysis

**DOI:** 10.1097/MD.0000000000024219

**Published:** 2021-01-22

**Authors:** Xiaorong Cheng, Shunqin Mao, Yibao Zhang, Xiaoyun Peng, Rui Ma, Yingcun Bao, Qun Li, Mei Liu, Dengjuan Sun, Bo Wan, Lulu Wang, Fang Zhang

**Affiliations:** Department of Rehabilitation Medicine, Second Hospital of Lanzhou University, Lanzhou, China.

**Keywords:** early physical rehabilitation, intracerebral hemorrhage stroke, rehabilitation, systematic review

## Abstract

**Background:**

The intracerebral hemorrhagic stroke (ICH) is associated with high mortality and severe disability in survivors, which causing about 42% of the disability-adjusted life years lost and 50% of all stroke patients dead within 1 year. Although early functional training is recommended to facility rehabilitation after the stroke, the benefit and safety are still controversial.

**Introduction:**

This systematic review aims to investigate whether early physical rehabilitation could have a beneficial effect for the patients with ICH compared with standard rehabilitation care.

**Methods and analysis:**

Pubmed, Embase, and Cochrane library will be searched to include randomized control trials which investigate the rehabilitation effective of the early mobilization for patients with ICH compared with routine nursing or standard care. Rev-Man version 5.3 will be used to perform all calculations related to the meta-analysis. Dichotomous data will be calculated in terms of a fixed or random effect model and expressed by the relative risk (RR) with 95% confidence interval (CI). The Cochrane collaborations tool in the following aspects was used to assess the risk of bias (ROB) in included studies. The inconsistency index (*I*^*2*^) and Chi-Squared will be applied for heterogeneity detection between clinical trials. A value of *P* < .05 will be considered statistically significant.

**Conclusion:**

This study will explore the role of early physical rehabilitation and provide insight for clinicals to improve rehabilitation results of ICH.

**Registration number:**

INPLASY2020110068.

## 1 Introduction

Stroke is one of the main factors leading to major disability and death in most countries in recent years, which reported that more than 795,000 people are affected in America.^[1]^ According to the clinical features and brain imaging, it is divided into 3 different types -- transient ischemic attack, ischemic stroke and hemorrhagic stroke. The hemorrhagic stroke is caused by leaking or bursting of the blood vessel, which account for about 20% of all strokes.^[2]^ The intracerebral hemorrhagic stroke (ICH) is associated with high mortality and severe disability in survivors,^[3,4]^ which causing about 42% of the disability-adjusted life years lost^[5]^ and 50% of all stroke patients dead within 1 year.^[6]^

Early functional training is recommended to facility rehabilitation after the stroke.^[7–9]^ However, the optimal initial rehabilitation time of functional activity is not clear. Several studies indicated that early physical rehabilitations might have a benefit for the rehabilitation among the patients with ICH.^[10–12]^ One study by Hsiao-Ching Yen etc.^[10]^ suggested that the early out-of-bed mobilization whin 24 to 72 hours might improve the functional independence compared with the standard rehabilitation (in-bed training). Ning Liu etc.^[13]^ conducted a multicenter, randomized controlled study compared early physical rehabilitation starting within 48 hours with the standard care group commencing rehabilitation after 7 days. They showed that early physical rehabilitation within 48 hours had a beneficial effect for the patients with ICH. Moreover, previous researches demonstrated that very early mobilization rehabilitation could increase the risk of bleeding again and cause worse outcomes.^[14–16]^ It is still controversial whether the early exercise is beneficial and safe for ICH. Therefore, this systematic review aims to explore whether early physical rehabilitation has a better effect for the patient with ICH than standard rehabilitation care.

## 2 Methods

This protocol was registered with the International Platform of Registered Systematic Review and Meta-Analysis Protocols (INPLASY, https://inplasy.com/) on November 17, 2020 (registration number INPLASY2020110068, https://inplasy.com/inplasy-2020–11-0068/).^[17]^ This review will develop following the Preferred Reporting Items for Systematic Reviews and Meta-Analyses (PRISMA) statement guidelines.^[18]^

### 2.1 Search strategy

A systematic search of the literature will be conducted using the PubMed, Web of science, Cochrane library, and 4 Chinese databases, which including Chinese Biomedical Databases (CBM), China National Knowledge Infrastructure (CNKI), Wanfang and Chongqing VIP. No restrictions in language, publication date or publication year are applied. Additional source including WHO clinical trial registry website, clinicaltrail.gov, conference abstracts, will also be searched. Further, the references of included trails will also be checked for more potential studies. The search strategy will use keywords and mesh term including “stroke”, “early physical rehabilitation”, “intracerebral hemorrhage”, and “early mobilization”, etc. The selection process will be presented in a PRISMA flow diagram (Fig. 1).

**Figure 1:** Flow diagram of study selection process.

### 2.2 Eligibility criteria

The RCTs which investigate the rehabilitation effective of the early mobilization for ICH compared with routine nursing or standard care will be eligible for this systematic review.

#### 2.2.1 Participants or population

Adult patients with ICH.

#### 2.2.2 Intervention

Early physical rehabilitation therapy starting within 72 hours of stroke onset.

#### 2.2.3 Comparator

Standard rehabilitation care.

#### 2.2.4 Study design

Only randomized controlled trials (RCTs) will be included.

#### 2.2.5 Main outcomes

The primary outcomes include the mortality, the functional performance and quality of life evaluated by the Functional Independence Measure (FIM-motor), Postural Assessment Scale for Stroke Patients, and Functional Ambulation Category (FAC), Modified Barthel Index, Short Form-36 (SF-36), and other validated scales. The secondary outcomes include the length of stay, recurrent stroke, and adverse effects.

### 2.3 Literature selection and data extraction

The retrieved records will be imported into the EndNote X9 software and the duplicate publications were excluded. Two reviewers independently read the titles and abstracts of all identified records to exclude those that are clearly not relevant. Then the full texts of the articles retained are reviewed to further determine their eligibility. Differences opinions were resolved by consensus.

The data are extracted by 2 reviewers independently using a pre-defined form. The following characteristics of included studies are collected: the first author, publication year, country, number of included patients, age, the detail of the intervention, treatment duration, follow-up time, and adverse events. Any discrepancies are resolved by consensus.

### 2.4 Quality assessment

The risk of bias (ROB) for included studies will be assessed using the Cochrane collaborations tool by 2 independent reviewers form the following dominants: the assessment includes sequence generation; allocation concealment; blinding of participants, personnel, and outcome assessors; incomplete outcome data; selective outcome reporting; and other sources of bias. Any differences between the authors on the data extraction and quality assessment will be resolves by discussion.

### 2.5 Strategy of data synthesis

Rev-Man version 5.3 will be used to conduct all calculations related to the meta-analysis. Dichotomous data will be calculated in terms of a fixed or random effect model and expressed by the relative risk (RR) with 95% confidence interval (CI). Continuous data will be presented as mean difference and 95% CI. The inconsistency index *(I*^*2*^) and Chi-Squared will be calculated for heterogeneity detection between studies. When assessing the difference in outcome, heterogeneity involving all trials will be examined. A value of *P* < .05 will be considered statistically significant. Egger test will be calculated to detect publication bias if there are at least ten studies included.

### 2.6 Subgroup analysis

The subgroup will be performed based on the several participants characters (including the various severity of stroke and different age), and therapy duration and start time of intervention, and the studies qualities according to the assessment results of risk of bias, etc.

### 2.7 Sensibility analysis

Sensitivity analysis will be carried out for primary outcomes by removing 1 study a time to investigate the robustness of the meta-analysis result.

## 3 Discussion

ICH is an important public health problem leading to high rates of death and disability in adults. It is crucial that commencing functional rehabilitation interventions as soon as possible to decrease disability caused by disease, meanwhile making sure the safety to avoid potential further damage for the ICH. More high-quality evidence focusing on the special schedule of early physical rehabilitation are needed to provide relevant reliable evidence to support the clinical practice.

## Author contributions

**Conceptualization:** Fang Zhang.

**Data curation:** Yibao Zhang, Xiaoyun Peng, Bo Wan, Lulu Wang.

**Formal analysis:** Shunqin Mao, Bo Wan, Lulu Wang.

**Investigation:** Shunqin Mao, Mei Liu, Dengjuan Sun.

**Methodology:** Xiaorong Cheng, Shunqin Mao, Rui Ma, Yingcun Bao, Qun Li, Mei Liu.

**Project administration:** Rui Ma, Qun Li.

**Software:** Xiaoyun Peng, Yingcun Bao, Dengjuan Sun.

**Supervision:** Fang Zhang.

**Visualization:** Yibao Zhang.

**Writing – original draft:** Xiaorong Cheng, Yibao Zhang.

**Writing – review & editing:** Yingcun Bao.
